# No Observed Effect of Landscape Fragmentation on Pathogen Infection Prevalence in Blacklegged Ticks (*Ixodes scapularis*) in the Northeastern United States

**DOI:** 10.1371/journal.pone.0139473

**Published:** 2015-10-02

**Authors:** Christine P. Zolnik, Richard C. Falco, Sergios-Orestis Kolokotronis, Thomas J. Daniels

**Affiliations:** 1 Department of Biological Sciences, Fordham University, Bronx, New York, United States of America; 2 Vector Ecology Laboratory, Louis Calder Center-Biological Field Station, Fordham University, Armonk, New York, United States of America; 3 New York State Department of Health, Louis Calder Center, Armonk, New York, United States of America; University of Maryland, College Park, UNITED STATES

## Abstract

Pathogen prevalence within blacklegged ticks (*Ixodes scapularis* Say, 1821) tends to vary across sites and geographic regions, but the underlying causes of this variation are not well understood. Efforts to understand the ecology of Lyme disease have led to the proposition that sites with higher host diversity will result in lower disease risk due to an increase in the abundance of inefficient reservoir species relative to the abundance of species that are highly competent reservoirs. Although the Lyme disease transmission cycle is often cited as a model for this “dilution effect hypothesis”, little empirical evidence exists to support that claim. Here we tested the dilution effect hypothesis for two pathogens transmitted by the blacklegged tick along an urban-to-rural gradient in the northeastern United States using landscape fragmentation as a proxy for host biodiversity. Percent impervious surface and habitat fragment size around each site were determined to assess the effect of landscape fragmentation on nymphal blacklegged tick infection with *Borrelia burgdorferi* and *Anaplasma phagocytophilum*. Our results do not support the dilution effect hypothesis for either pathogen and are in agreement with the few studies to date that have tested this idea using either a landscape proxy or direct measures of host biodiversity.

## Introduction

The northeastern and upper Midwestern United States experience the highest densities of blacklegged ticks (*Ixodes scapularis* Say, 1821) [1, 2] and consequently report the highest rates of human cases for associated tick-borne diseases, annually [3]. However, the prevalence of tick-borne pathogens in blacklegged tick populations varies considerably across these regions, even within areas where the tick and its pathogens are well established [4–9]. A large body of research exists identifying suitable habitats for blacklegged ticks, as well as environmental and climatic factors that influence the spatial distribution and the increase and spread of these populations [2, 10–14]. However, there is less of a consensus regarding the factors that influence tick infection prevalence and disease risk. A widely reported hypothesis for the variation in tick infection rates with the Lyme disease pathogen (*Borrelia burgdorferi*) is the “dilution effect”. This hypothesis proposes that at sites with higher host species diversity, an increase in the relative abundance of inefficient reservoirs and a subsequent decrease in the relative abundance of a highly competent reservoir (i.e., white-footed mouse, *Peromyscus leucopus*), will result in a decrease in tick infection prevalence [15–17].

Four characteristics have been deemed necessary for the dilution effect to work in a vector-borne disease system: (1) a generalist vector, (2) oral acquisition of the pathogen, and (3) variation in host reservoir competence with (4) the most competent reservoirs being dominant in the community [15]. Although the Lyme disease system appears to meet all of these assumptions, most studies examining the dilution effect with respect to Lyme disease have relied on computer simulation models with input from limited field-collected data [15–19]. These studies often use large spatial scales (e.g., state level) to tally species richness as a measure of diversity [16, 20]. Using large spatial scales has inherent problems, as the variables (i.e., species richness) can vary widely across large geographic areas. Additionally, averaging over a large area does not necessarily take into account the influence of local factors, or local disease risk. Overlooking potentially informative local scale variation makes these models overly generalized. Furthermore, many of these studies use human Lyme disease incidence as their risk measure [16, 20]. Human case data are based on confirmed cases, which require the presence of a number of clinical criteria [21]. A recent report presented by the CDC estimates actual number of Lyme cases to be as much as 10 times greater than the reported cases on an annual basis [22]. Furthermore, human Lyme disease case data are based on patient residence location, rather than the location where the infected tick was acquired, which can lead to misinterpretation of the real risk at a particular site.

Host biodiversity at a particular site is often a difficult measure to attain. For example, trapping time, manpower, equipment, and supplies needed to sample a wide range of animals are usually limited. Additionally, some hosts are more easily captured and the range of species collected tends to be biased for larger animals that are easier to see and handle, thus, trapping effort across animal taxa is highly uneven. Each of these deficiencies can bias both species richness and abundance data. As blacklegged ticks have a wide host range of more than 120 potential vertebrate species [23], true estimates of biodiversity of potential hosts are very difficult to assess. This difficulty has led some studies to infer levels of biodiversity based on certain habitat features. For instance, many studies find patterns of decreasing biodiversity with increasing habitat fragmentation [24–29]. With respect to tick-borne disease systems, two studies have attempted to determine the influence of forest fragmentation –as a proxy for host biodiversity– on measures of blacklegged tick infection and density, finding increasing infection prevalence in ticks at sites with higher fragmentation [30, 31]. However, both studies were limited by the number of ticks tested at each site (average 20–25). Additionally, Brownstein et al. [31] used adult tick infection prevalence for their analyses, but it is unclear how this measure for adult ticks relates to human risk.

The goal of this study was to determine the effect of landscape fragmentation on nymphal infection prevalence (NIP) and density of infected nymphs (DIN) in a region of the Unites States where the tick vector is well established and its associated pathogens are endemic [1, 2]. Our study focused on nymphs, as this tick developmental stage is responsible for the vast majority of human Lyme disease cases [32]. Although a number of studies use NIP as a measure of human disease risk [18, 19, 33], the density of infected nymphs is considered the most direct risk measure to humans (entomological risk) [34]. Specifically, we used forest patch size and percent impervious surface, both as measures of forest fragmentation (a proxy for host biodiversity), to explore this relationship on NIP and DIN. We determined the effect of these landscape fragmentation variables on the prevalence of nymphal ticks infected with *Borrelia burgdorferi* and *Anaplasma phagocytophilum*. Lyme disease is the most common vector-borne disease in the United States [3] and its causative agent *B*. *burgdorferi* is more prevalent in tick and host populations than *A*. *phagocytophilum*. However, the incidence of its associated disease, human granulocytic anaplasmosis, has been increasing in recent years [35], and it is well-established in tick populations in areas where *B*. *burgdorferi* is prevalent [4–9]. If host biodiversity influences NIP or DIN of *B*. *burgdorferi*, it should likewise influence these risk measures with *A*. *phagocytophilum*, as both pathogens share the same tick vector, route of pathogen acquisition, and dominant reservoir host (white-footed mouse) [36–40].

## Materials and Methods

### Site Selection and Classification

Fourteen forested sites along a 115-km urban-to-rural gradient were selected for this study [41]. This urban-to-rural gradient runs from New York City to rural western Connecticut [41] and sites for this study were located within three counties in southern New York (Bronx, Westchester, and Putnam) and one county in western Connecticut (Litchfield) (Fig 1). Bronx and southern Westchester counties have forests that are heavily fragmented and a comparatively large fraction of the land is covered with impervious surface. This fragmentation and imperviousness decreases into northern Westchester, Putnam and Litchfield counties [41]. Blacklegged ticks in this region are highly prevalent and the area is endemic for both *B*. *burgdorferi* and *A*. *phagocytophilum* [1, 2, 7, 42]. All sampling sites were located in state, county, or city public lands and were comprised of deciduous forest cover; sampling locations were at least 7.5 km from each other. Appropriate scientific collection permits were obtained from all relevant agencies.

**Fig 1:** Tick collection localities in New York and Connecticut. Locations of the fourteen sampling sites used in this study across four counties in southern New York and western Connecticut with land cover types from the 2011 National Land Cover Database (NLCD) [43]. Site locality information is consistent with Table 1. Site markers are not drawn to scale. Inset shows a map of the region at state level for reference. Box indicates magnified area.

As dispersal of blacklegged ticks are primarily accomplished via host movement, and pathogen acquisition is from the bloodmeal of a competent reservoir, the impact of forest fragmentation on populations of this tick was studied at the typical home ranges of three types of hosts. Three buffers (100, 400, 1000-m radii) were created around each sampling center point representing the typical home ranges of small- (i.e., white-footed mice), medium- (i.e., raccoons, *Procyon lotor*) and large-bodied (i.e., white-tailed deer, *Odocoileus virginianus*) hosts, respectively [44–47]. Although home ranges can vary both temporally and spatially, these buffers were used to represent typical home ranges during the summer months, when tick collection was conducted, for statistical purposes. Within each buffer, average impervious surface was determined using zonal analysis in ArcGIS v10.1 (ESRI) on the 2011 Percent Developed Imperviousness shapefile from the USGS National Land Cover Data [48]. All data from the NLCD were collected at a 30-m resolution.

To determine the forest patch size for each sampling site, forested areas were selected from the NLCD 2011 Land Cover layer [43]. Forested areas were considered part of a forest patch if located at least 200 m from the next forested area. This distance represents the typical home range of small hosts (i.e., white-footed mouse), and would therefore likely be the minimum distance these ticks are dispersed on hosts. Due to the lack of isolated forested patches for 11 sites, we attempted a more conservative distance criterion of 100 m, but also found that the lack of isolated forested patches persisted for those 11 sites.

### Tick Collections and Pathogen Testing

In June and July 2013, nymphal blacklegged ticks were collected from an area of at least 1000 m^2^ at each of the 14-forested sites by dragging with a 1-m^2^ cloth along the forest floor in 20 m transects. After each transect, ticks were counted and collected before being transported back to the lab for species and life stage identification. All ticks were stored at -80°C until further processing.

Small sample sizes may preclude accurate assessments of true infection rates in ticks. Consequently, we attempted to determine the minimum number of ticks needed to accurately calculate the infection rate in nymphs. We set a “true” population of 100 ticks with an infection rate of 25% and conducted bootstrap resampling with replacement for a variety of sample sizes, ranging from 10 to 55 ticks at intervals of 5, with 1,000 iterations at each interval (Resampling Stats for Excel, statistics.com LLC, Arlington, VA). An infection rate of 25% was chosen as representative of the mean infection with *B*. *burgdorferi* in northeastern *I*. *scapularis* populations [5, 7]. In addition to the infection rate for each of the samples, the overall mean infection rate, the variance, the coefficient of variation, and 95% confidence intervals were calculated for the entire set of estimates at each of the 10 sample sizes (e.g., 10, 15, 20, 25…55 nymphs). Data were plotted graphically and we found that (1) the variance declined through a sample size of 35 ticks and stabilized at 40 ticks and higher, (2) the coefficient of variation declined through a sample size of 30 ticks and stabilized between 35 and 40 ticks, and (3) the confidence intervals narrowed through a sample size of 40 ticks and became stable after that. These analyses suggest that a conservative minimum sample size of 40 nymphs would be needed before an estimate of infection rate that approaches the true infection rate could be obtained. However, further analyses of the frequency distribution of individual infection rate estimates at each sample size indicate that the likelihood of obtaining an accurate infection rate, defined in this experiment as one between 20% and 30% (i.e., within 5% of the true infection rate) was just about 1 in 4 for samples of less than 40 nymphs, 1 in 2 for samples of 50 nymphs, but 3 in 4 for samples of 55 nymphs. Based on the frequency distributions, we determined that sampling at least 55 nymphs per site would optimize chances of obtaining an accurate estimate of the infection rate while balancing the need to sample all sites in the limited nymphal activity period. Thus, we tested a total of 56 nymphal ticks for each site.

DNA extractions were performed on bisected nymphs using the DNeasy Blood & Tissue Kit (QIAGEN), with an overnight incubation at 56°C in ATL lysis buffer and proteinase K, and a final elution in 100 μl ddH_2_O. Each tick was tested in triplicate for *B*. *burgdorferi* and *A*. *phagocytophilum* using a duplex quantitative real-time PCR (referred to as qPCR) assay protocol with absolute quantification developed by Courtney et al. [49]. This protocol tests for a *B*. *burgdorferi*-specific 75-bp fragment of the 23S rRNA gene and an *A*. *phagocytophilum*-specific 77-bp fragment of the *msp2* gene. We used 12.5 μl of 2× TaqMan Universal Master Mix II (Applied Biosystems, Inc.), 1.25 μl of ddH2O, primers ApMSP2f / ApMSP2r and Bb23Sf / Bb23Sr at final concentrations of 0.9 μM and 0.7 μM each, respectively, and probe ApMSP2p-VIC and probe Bb23Sp-FAM at final concentrations of 0.125μM and 0.175μM, respectively [49]. Thermal cycling conditions were 50°C for 2 min, 95°C for 10 min, and 40 cycles of 95°C for 15 s, followed by 60°C for 60 s with a plate read after each cycle. All pathogen testing was performed on an ABI 7300 Real-Time PCR System (Applied Biosystems, Inc.).

### Statistical Analysis

Nymphal infection prevalence (NIP) was recorded as the number of ticks infected with each pathogen at each site (n = 56). A Spearman’s rank order correlation was conducted to determine if *B*. *burgdorferi* and *A*. *phagocytophilum* were correlated in prevalence. Density of infected nymphs per 1000 m^2^ (DIN) was determined by multiplying the NIP by the density of nymphs per 1000 m^2^ at each site (DON).

To determine the influence of the landscape variables on the prevalence of each pathogen, we fit negative binomial regression models to the number of infected nymphal blacklegged ticks per site, and the density of infected nymphs using average impervious surface as the predictor value for both models. Because disease data tend to be overdispersed, a negative binomial distribution applies [50]. We applied separate models for each pathogen (*B*. *burgdorferi* and *A*. *phagocytophilum*) and dependent value (NIP and DIN) at each buffer size, and the overall model fit for each was determined using a *χ* ^2^ goodness-of-fit test. Due to the lack of isolated forested patches for 11 of the 14 sample sites, forest patch size was not included in these models.

To determine if pathogen prevalence was distributed randomly among the 14 collection locations, we performed an autocorrelation using Global Moran’s *I* for each pathogen. All statistics were considered significant at *P <* 0.05 and data analyses were conducted in R 3.1.2 [51]. Spatial analysis was performed in ArcGIS v10.1 (ESRI). All spatial data were projected to NAD 1983-18N.

## Results

A total of 784 nymphal ticks (56 ticks from each of the 14 sites) were tested for *B*. *burgdorferi* and *A*. *phagocytophilum* using qPCR TaqMan assays. Thirteen sites had at least one tick positive for *B*. *burgdorferi* and six sites had at least one tick positive for *A*. *phagocytophilum* (Table 1). Only one site showed coinfection with both pathogens. Overall NIP with *B*. *burgdorferi* ranged from 0 to 33.9% (mean = 17, SE = 2.46) and with *A*. *phagocytophilum* ranged from 0 to 14.3% (mean = 2.7, SE = 1.21) (Table 1). Density of nymphs (DON) ranged from 27 to 140 ticks per 1000 m^2^ and DIN ranged from 0 to 23.68 (mean = 12.89, SE = 2) for *B*. *burgdorferi* and 0 to 8.28 (mean = 1.92, SE = 0.79) for *A*. *phagocytophilum* (Table 1).

**Table 1:** Collection locality and sample information.

Site	Town	County, State	DON	*B*. *burgdorferi*		*A*. *phagocytophilum*	
				NIP	DIN	NIP	DIN
A	Bronx	Bronx, NY	34	26.79%	9.11	0.00%	0.00
B	Yonkers	Westchester, NY	133	16.07%	21.38	0.00%	0.00
C	Rye	Westchester, NY	31	12.50%	3.88	0.00%	0.00
D	Armonk	Westchester, NY	140	10.71%	15.00	3.57%	5.00
E	Ossining	Westchester, NY	46	0.00%	0.00	10.71%	4.93
F	Cortlandt	Westchester, NY	78	7.14%	5.57	0.00%	0.00
G	Katonah	Westchester, NY	75	25.00%	18.75	0.00%	0.00
H	Bedford	Westchester, NY	110	14.29%	15.71	0.00%	0.00
I	Pound Ridge	Westchester, NY	89	16.07%	14.30	1.79%	1.59
J	North Salem	Westchester, NY	68	12.50%	8.50	0.00%	0.00
K	Carmel	Putnam, NY	78	30.36%	23.68	0.00%	0.00
L	Kent	Litchfield, CT	27	17.86%	4.82	1.79%	0.48
M	Sharon	Litchfield, CT	125	16.07%	20.09	5.36%	6.70
N	Goshen	Litchfield, CT	58	33.93%	19.68	14.29%	8.29

Location of each site and density of nymphs per 1000 m^2^ (DON), nymphal infection prevalence (NIP), and density of infected nymphs per 1000 m^2^ (DIN) for both *B*. *burgdorferi* and *A*. *phagocytophilum*

Prevalence of the two pathogens was not correlated (Spearman’s r_S_ = -0.02, *P* = 0.95). Spatial autocorrelation demonstrated that nymphal infection prevalence for each pathogen was randomly distributed across the fourteen sites (Moran’s *I z*-score = 0.26, *P* = 0.80).

We required forested land cover to be at least 200 m from the next forested area in order to be considered an isolated forest patch. Only three of our sample sites were found to be isolated from one another while 11 sites were determined to be located within contiguous forest cover. This pattern was also observed when a more conservative criterion of 100 m was used. The three isolated forest patches ranged in size from 0.36 to 0.77 km^2^ (mean = 0.53, SE = 0.13) when using the 200 m criterion, and from 0.40 to 1.87 km^2^ (mean = 1.07, SE = 0.43) when using the 100 m criterion. Due to the limited number of sample sites located within isolated forest patches, this variable was not used in the negative binomial regression model. Average percent impervious surface within the three buffer levels (100, 400, 1000 m) around each site ranged from 0 to 20%. To determine the relationship between nymphal infection prevalence and impervious surface, a negative binomial regression model was used. No significant relationship between percent impervious surface and nymphal infection prevalence with either pathogen was found at any of the three buffer levels. Similarly, there was no significant relationship between percent impervious surface and density of nymphs infected with *B*. *burgdorferi* (Table 2) or with *A*. *phagocytophilum* (Table 3).

**Table 2:** Regression analysis results for *Borrelia burgdorferi*.

		Estimate	SEM	*z*-value	*P*
**NIP**	Intercept	2.281	0.171	13.353	<0.0001
	100m Buffer	-0.019	0.066	-0.289	0.772
	Intercept	2.312	0.177	13.068	<0.0001
	400 m Buffer	-0.020	0.035	-0.588	0.557
	Intercept	2.348	0.175	13.432	<0.0001
	1000 m Buffer	-0.022	0.022	-0.978	0.328
**DIN**	Intercept	2.484	0.206	12.084	<0.0001
	100m Buffer	0.044	0.076	0.571	0.568
	Intercept	2.532	0.219	11.547	<0.0001
	400 m Buffer	0.004	0.041	0.092	0.926
	Intercept	2.607	0.219	11.901	<0.0001
	1000 m Buffer	-0.015	0.027	-0.566	0.571

Results from negative binomial regression models for nymphal infection prevalence (NIP) and density of infected nymphs per 1000 m^2^ (DIN) of *B*. *burgdorferi* and the predictor value of average impervious surface within three buffers (100, 400, 1000 m) around each site.

**Table 3:** Regression analysis results for *Anaplasma phagocytophilum*.

		Estimate	SEM	*z*-value	*P*
**NIP**	Intercept	0.750	0.575	1.304	0.192
	100m Buffer	-0.521	0.534	-0.975	0.330
	Intercept	0.994	0.516	1.925	0.054
	400 m Buffer	-0.622	0.386	-1.613	0.107
	Intercept	0.905	0.497	1.821	0.069
	1000 m Buffer	-0.309	0.202	-1.529	0.126
**DIN**	Intercept	0.985	0.577	1.708	0.088
	100m Buffer	-0.357	0.357	-1.000	0.317
	Intercept	1.256	0.550	2.285	0.022
	400 m Buffer	-0.461	0.281	-1.641	0.101
	Intercept	1.202	0.528	2.278	0.023
	1000 m Buffer	-0.241	0.139	-1.730	0.084

Results from negative binomial regression models for nymphal infection prevalence (NIP) and density of infected nymphs per 1000 m^2^ (DIN) of *A*. *phagocytophilum* and the predictor value of average impervious surface within three buffers (100, 400, 1000 m) around each site.

## Discussion

Our sampling area represents a region of the northeastern United States with well established populations of *I*. *scapularis* and a relatively high prevalence of *B*. *burgdorferi* and *A*. *phagocytophilum* in tick populations [1, 2, 7, 42]. Despite this, infection prevalence in tick populations differs among sites in this area [4–9], a finding that our results support. Previous studies have suggested that variation in infection rates for Lyme disease is due to different levels of host biodiversity, as proposed by the dilution effect hypothesis [15–17]. However, we found no evidence to support the dilution effect for the Lyme disease pathogen when using level of urbanization as a proxy for biodiversity. Our results also did not support the dilution effect for *A*. *phagocytophilum*, and, although this pathogen has not been studied with respect to the dilution effect, its vector, reservoir hosts, and pathogen transmission route are the same as for *B*. *burgdorferi*.

A previous study investigating the relationship between tick infection prevalence and habitat patch size used patches with mean isolation distances ranging from 0 to 134.2 m [31]. These short distances are unlikely to limit most host movements, and, therefore, are unlikely to constitute discreet forested patches in which infection prevalence can be analyzed separately. Allan et al. [30] sampled within sites that were at least 1.6 km from the nearest forested area and identified a 2-ha threshold, below which density of infected nymphal ticks was higher than in larger patches. However, as pointed out in a recent review by Randolph and Dobson [52], patches less than 2 ha are too small for resident populations of white-tailed deer, which are crucial for maintaining populations of this tick species [53–57], and care should be taken when extrapolating the dilution effect hypothesis to a more generalized landscape. Furthermore, the small average sample size of ~20 nymphal ticks tested for *B*. *burgdorferi*, limits the ability to accurately assess infection prevalence at each site. Due to the limitation in tick sample size for both of these studies, as well as the limited isolation of some of the patches in Brownstein et al. [31], the need for studies that quantify the effect of habitat patch size on measures of disease risk is warranted. Our current study demonstrates the difficulty in assessing habitat patch size that are suitable for tick populations in suburban and rural areas, as we were unable to determine the effect of forest patch size on measures of disease risk due to the limited number of isolated forested patches.

Since the dilution effect hypothesis is based on host biodiversity, the ideal test would be to determine the effect of host biodiversity directly on measures of disease risk, NIP or DIN. However, there are limited studies that have explored this relationship directly [33, 58]. LoGiudice et al. [33] found a significant negative relationship between host species richness and NIP across 37 habitat fragments, but a large number of the sites (n = 12, 32.4%) had <30 ticks (of which four fragments had <5 ticks), on which to determine NIP. Estimating NIP with so few ticks should be done cautiously. When LoGiudice et al. [33] examined their data using only patches with at least 30 nymphal ticks (n = 26 fragments), no significant relationship between host species richness and NIP was found. Recently, States et al. [58] reported a lack of support for the dilution effect hypothesis between species-poor and species-rich vertebrate communities (island vs. mainland) for sites where host biodiversity was directly measured.

As studies and reviews begin to question the validity of the dilution effect as a basis for understanding blacklegged nymphal infection prevalence and/or density of infected nymphs and consequently Lyme disease risk to humans [52, 58–60], it is becoming clear that the ecological factors affecting site-to-site variation in infection rates are still largely unknown. Thus, additional research is warranted and possible factors that should be explored further include the influence of host immunity and host community composition, as opposed to host biodiversity as a whole, as well as variation in pathogen strains, which may influence pathogenicity or dissemination in a host. It is also possible that internal factors are influencing pathogen infection within populations of these ticks. For example, Hersh et al. [61] found co-infections rates with *Babesia microti* and *B*. *burgdorferi* higher than expected due to chance alone. It has been suggested that *B*. *microti* acquisition by *I*. *scapularis* may be promoted by infection with *B*. *burgdorferi* [62], a factor that may explain variation in infection with either or both of these two pathogens across sites. In this study, no correlation was found between the prevalence of *B*. *burgdorferi* and *A*. *phagocytophilum*, and only one site had coinfections with both pathogens. Another study did not find an interaction effect between *B*. *burgdorferi* and *A*. *phagocytophilum* in ticks, and that study demonstrated that the presence of one of these agents in a tick did not affect the acquisition of the other from a host [63]. It is unlikely that these particular two pathogens play a large role together in terms of the variation of NIP or DIN observed in nature. However, little is known regarding the identity of non-pathogenic microorganisms, and how individual microorganisms, or microbial communities, may influence the acquisition, maintenance, or removal of pathogens within these ticks. Further investigation into the identity of the microbial communities present in this tick species and the potential correlations between overall microbial diversity and known tick-borne pathogens will shed light on the possible influence that internal microbial structure has on this tick and tick-borne pathogens.

## Conclusions

The dilution effect hypothesis states that biodiversity within a community can act as a buffer against infectious disease risk by effectively decreasing the relative abundance of a few highly competent reservoir species compared to the relative abundance of inefficient reservoirs. Over the past 15 years, the Lyme disease transmission cycle has frequently been cited as a model supporting this hypothesis, despite limited empirical data. Recent studies have begun to question the validity of the dilution effect hypothesis [52, 58, 59], however, and the current study—an examination of blacklegged tick pathogen prevalence across an urban-to-rural landscape gradient in southern NY and western CT states—further undermines claims that the dilution effect has any role in explaining Lyme disease risk.

In light of growing evidence refuting the dilution effect hypothesis with respect to Lyme disease risk, future studies should investigate factors other than biodiversity including host and reservoir community composition beyond the dominant species and how that changes from year-to-year. Long-term ecological studies will provide insight into factors affecting changes in infection prevalence and tick abundance. It is becoming increasingly clear that biodiversity per se does not provide the buffer against Lyme disease risk that has been suggested by studies advocating the dilution effect hypothesis. Furthermore, intraspecific mechanisms within the tick vector deserve a closer examination. In an era of high-throughput sequencing that allows researchers to investigate genome-wide effects of host immunity microevolution on tick-borne pathogens, as well as the virulence of different pathogen strains, limiting studies to such broad topics as ‘biodiversity’ may only serve to obstruct our understanding of actual causative factors.
